The article "DNA Methyltransferase Inhibitor 5-AZA-DC Regulates TGFβ1-Mediated Alteration of Neuroglial Cell Functions after Oxidative Stress" was retracted in 2023. Reasons: signs of a paper mill; compromised peer review; unreliable results or conclusions.

# DNA Methyltransferase Inhibitor 5-AZA-DC Regulates TGF*β*1-Mediated Alteration of Neuroglial Cell Functions after Oxidative Stress

**DOI:** 10.1155/2022/9259465

**Published:** 2022-09-28

**Authors:** Xiao-Yong Zhao, Xiao-Li Zhang

**Affiliations:** ^1^Department of Neurosurgery, Affiliated Huadu Hospital, Southern Medical University (People's Hospital of Huadu District), Guangzhou 510800, China; ^2^The Third School of Clinical Medicine Southern Medical University, Guangzhou, China; ^3^Department of Neurosurgery, Affiliated Fifth Hospital, Guangzhou Medical University, Guangzhou, China; ^4^Department of Obstetrics and Gynecology, Affiliated Huadu Hospital, Southern Medical University (People's Hospital of Huadu District), Guangzhou 510800, China; ^5^Department of Obstetrics and Gynecology, The Second People's Hospital of Guangdong Province, Guangzhou, China

## Abstract

5-AZA-DC is an efficient methylation inhibitor that inhibits methylation of target DNA. In this study, we explored the effects of 5-AZA-DC on the regulation of TGF*β*1 on target genes in neuroglial cell, as well as neuroglial cell functions under oxidative stress. The oxidative stress was constructed by editing CRISPR/Cas9 for knock out Ang-1 and ApoE4 genes. Cells were subjected to TGF*β*1^OE^ (or shTGF*β*1) transfection and/or 5-AZA-DC intervention. Results showed that under oxidative stress, both TGF*β*1^OE^ and shTGF*β*1 transfection raised DNMT1, but reduced TGF*β*1, PTEN, and TSC2 expressions in neuroglial cells. TGF*β*1 directly bind to the promoter of PTEN gene. 5-AZA-DC intervention lowered DNMT1 and raised TGF*β*1 expression, as well as promoted the binding between TGF*β*1 and promoter of PTEN. TGF*β*1^OE^ caused a significant increase in the DNA demethylation level of PTEN promoter, while 5-AZA-DC intervention reduced the DNA demethylation level of PTEN promoter. Under oxidative stress, TGF*β*1^OE^ (or shTGF*β*1) transfection inhibited neuroglial cell proliferation, migration, and invasion, promoted cell apoptosis. 5-AZA-DC intervention alleviated TGF*β*1^OE^ (or shTGF*β*1) transfection caused neuroglial cell proliferation, migration, and invasion inhibition, as well as cell apoptosis. To conclude, these results suggest that 5-AZA-DC can be used as a potential drug for epigenetic therapy on oxidative stress damage in neuroglial cells. The findings of this research provide theoretical basis and research ideas for methylation drug intervention and TGF*β*1 gene as a possible precise target of glial oxidative stress diagnosis and treatment.

## 1. Introduction

Oxidative stress (OS) is a state of imbalance between oxidation and antioxidant effects in the body, which is caused by the increase of oxidative reactions and decrease of antioxidant reactions [1]. Lots of reactive oxygen species (ROS), including peroxides, superoxides, hydroxyl radical, single oxygen, and alpha-oxygen are produced in this process [2]. They can damage DNA, proteins and lipids in cells, thereby lead to injury of tissues [3].

Brain is the nerve center of human body. Oxidative stress is one of the most important pathological mechanisms of ischemic stroke and the main reason for irreversible cerebral ischemia/reperfusion injury [4]. Neuroglial cells are another type of cells other than neurons in neural tissue, including astrocytes, oligodendrocytes, and microglia cells [5]. Compared to neurons, neuroglial cells also have processes, but no dendrites and axons, which widely distributed in the central and peripheral nervous system and is fully involved in the tasks of neuronal information transmission and processing, as well as in maintaining microenvironmental homeostasis [5]. In mammals, the ratio of neuroglial cells to neurons is about 10 : 1. Previous literature reported that excessive ROS could cause rapid deterioration of neuroglial cell function [6]. Prevention of oxidative stress is considered as a critical pathway in the treatment of various intracranial diseases [4, 7].

Recent years, the relationship between DNA methylation and gene expression at the transcription level aroused more and more attention. It is demonstrated that alterations of DNA methylation, particularly the alteration within the regulatory regions of genes expression, significantly impacts on gene transcription [8]. Moreover, lots of studies discover that oxidative stress can cause epigenetic changes, especially influence DNA methylation level, in which hypermethylation can induce gene transcriptional repression and hypomethylation induce gene transcriptional activation [9, 10]. It is reasonable to assume that the injury of neuroglial cells caused by oxidative stress is associated with the change of DNA methylation induced gene expression alteration in cells [11]. The mechanism and clinical significance of epigenetic changes of oxidative stress, especially DNA methylation alteration in oxidative stress is still unclear [12, 13]. In our study, we firstly constructed the TGF*β*1 overexpressed and silenced neuroglial cell lines, and then applied 5-AZA-DC, an efficient methylation inhibitor, intervention to compare oxidative stress and normal neuroglial cell strain biological and functional differential through multiomics collaborative studies. Furthermore, we explored the function of the epigenetic regulatory molecule TGF*β*1 in oxidative stress of neuroglial cell. The findings of research will be not only useful for elucidating the regulatory mechanism of TGF*β*1 in oxidative stress, but also provide potential therapeutic targets and drugs for the targeted treatment of oxidative stress.

## 2. Materials and Methods

### 2.1. Cell Culture and Experimental Treatments

Neuroglial cell line HEB was purchased from the Cell Resource Center of Shanghai Academy of Life Sciences, Shanghai Academy of Biological Sciences (Shanghai, China). Neuroglial cell lines HM, HM06, and SVGP12 were purchased from American Type Culture Collection (ATCC, VA, USA). The culture of HEB and HM cells were cultured in RPMI-1640, while HM06 and SVGP12 cells were cultured in DMEM/F12. RPMI-1640 and DMEM/F12 were supplemented with 10% fetal bovine serum (FBS), 100 *μ*g/mL penicillin and 100 *μ*g/mL streptomycin. All cells were placed in an incubator of 37°C with 5% CO_2_.

### 2.2. Intracellular Knockout of Ang-1 and APOE4 Genes of Neuroglial Cells by CRISPR/cas9

Appropriately 2 × 10^7^ cells were taken to target the Ang-1 and APOE4 genes, appropriate targets were selected, and gene editing tools were designed using CRISPR/cas9 technology was applied to knockout the Ang-1 and APOE4 genes in about 2 × 10^7^ neuroglial cells. Appropriate targets were selected and the tools plasmid was transfected into cells. Gene knockout was achieved using the restriction effect after its expression. Each pair of guide oligo will be complementary connected. The ligated oligo mixture in the upper step was diluted with ddH_2_O in a 1 : 200 ratio at room temperature and oligo was ligated with the pSpcas9(BB)-2A-GFP plasmid. Plasmids were extracted and sequenced with U6 primers.

### 2.3. Establishment of Oxidative Stress Model in Oxyglucose Deprivation/Reoxygenic Astrocytes

Cells were growth in culture medium containing 10% FBS at 37°C with 5% CO_2_, the supernatant was discarded after centrifugation at 800rmp for 5 min. Then, 2 *μ*g transfected plasmid (sg RNA) was added to the transfection cup and electros pun in the T16 procedure. Following rinsed twice with PBS, cells were subjected to oxygen sugar deprivation: sugar-free culture medium, no FBS, 1% O_2_, 5% CO_2_, for 5 hours. Subsequently, cells were grown in reoxygenation condition culture: normal culture medium containing 10% FBS, 20% O_2_, and 5% CO_2_.

### 2.4. Establishment of TGF*β*1 Gene Overexpression and Silenced Cell Lines

After following hypoxic stimulation, about 1 × 10^5^ neuroglial cells in 500 *μ*L FBS-free culture medium were added into 24-well plate. 20 *μ*L target lentivirus (TGF*β*1-cDNA) or empty-load lentivirus was added into each well and incubated at 37°C for 48 h. Then, TGF*β*1 protein expression in cells was determined by western blot to identify the overexpression and silence of TGF*β*1. Cells without any treatment were set as blank control groups (Con group), cells subjected to Ang-1 and APOE4 knockout were divided into oxidative stress TGF*β*1 gene silencing group (shTGF*β*1 group) and oxidative stress TGF*β*1 overexpression group (TGF*β*1^OE^ group). The sequences of shTGF*β*1 and sh control were shown in Table 1.

### 2.5. DNA Methyltransferase Inhibitor (5-aza-2-deox-ycytidine, 5-AZA-DC) Treatment

After oxyglucose deprivation/reoxygenic stimulation, about 2 × 10^5^ cells from each group were seeded in 6-well plates overnight. Then, the fresh medium containing 5 *μ*M 5-AZA-DC (Sigma-Aldrich, MO, USA) was added into culture medium for 72 h. Blank control groups were treated with 0.01% DMSO culture medium.

### 2.6. Quantitative Real-Time PCR (qRT-PCR)

To test the mRNA expressions of DNMT1, TGF*β*1, PTEN, and TSC2, quantitative real-time PCR was conducted. After relevant treatment, cells were harvested in 1.5 mL EP tubes and 1.0 mL of Trizol solution was added for 5 min at room temperature. Then, 0.2 mL chloroform was supplemented into tube and tube was centrifuged at 4°C at 12000rmp for 15 min. Supernatant was discarded and 1 mL of 75% ethanol was added to wash RNA precipitate one time (centrifuged at 7500rmp for 5 min). RNA concentration was determined using a microamount RNA/DNA quantimeter. The relative expressions of DNMT1, TGF*β*1, PTEN, and TSC2 were detected using BeyoFast™ SYBR Green One-Step qRT-PCR Kit (Beyotime Biotechnology, Shanghai, China). The reaction conditions were set as: (1) 95°C for 10 min, (2) 40 cycles of 95°C for 5 s and 60°C for 30 s, (3) 94°C for 30 s, 60°C for 90 s, and 94°C for 10 s. Primer's information was displayed in Table 2. Data were analyzed using 2^-△△CT^ method and *β*-actin was served as internal control.

### 2.7. Western Blot

After relevant stimulation, cells were harvested, incubated with RIPA Lysis buffer, and fragmented by sonication on ice. Following centrifugation at 4°C, 12000 rpm for 30 min, the supernatant containing proteins was collected. BCA assay was carried out to measure protein concentration and equal concentration of proteins were subjected to electrophoresis and transferred onto polyvinylidene fluoride (PVDF) membrane, which were incubated with anti-TGF*β*1 antibody (1 : 1000, Thermo Fisher Scientific, PA5-36923), anti-PTEN antibody (1 : 1000, Thermo Fisher Scientific, PA5-90331), anti-DNMT1 antibody (1: 1000, Abclonal, AP0528), anti-TSC2 antibody (1: 1000, Abclonal, AP2662), and anti-*β*-actin antibody (1: 2000, Proteintech Group, #60011-3) overnight at 4°C. Subsequently, PVDF membrane was incubated with relevant secondary antibodies. Protein bands were visualized using ECL system and grayscale values of the bands were analyzed using Image-Pro Plus image software.

### 2.8. GST-Pull Down Assay

GST-pull down assay was carried out to confirm the interaction of TGF*β*1 with PTEN and TSC2. After relevant stimulation, cells were harvested, washed with PBS, and lysed on ice. Then, His-tag-TGF*β*1, GST-PTEN, and GST-TSC2 was mixed with cell lysates. In the group output samples, 20 *μ*L glutathione agarose beads were added. The glutathione agarose beads containing the GST empty protein were operated in parallel as control. Following boiled at 100°C for 5 min. Results were analyzed by western blot.

### 2.9. Chromatin Immunoprecipitation Assay (CHIP) Assay

CHIP assay was carried out to verify the direct binding effect of TGF*β*1 to the target gene PTEN. After relevant stimulation, cells were lysed using sonication breaker on ice and cell suspension was centrifuged at 4°C, 12000 rpm for 10 min. 10 *μ*L of the supernatant was taken as an input, and the remaining supernatant was supplemented with 2 *μ*g of the primary antibody and the corresponding rabbit IgG. Subsequently, 1 *μ*L RNase was added and incubated at 37°C for 30 min. The PCR products were separated by 2% agarose gel electrophoresis, then photographed and analyzed.

### 2.10. Dual-Luciferase Reporter Gene Assay

The gene sequence containing PTEN promoter was inserted into the upstream of pGL3-Basic/luciferase vector luciferase, designated as pGL3-PTEN-luc. Cell transfection was conducted using lipofectamine 2000. The luciferase fluorescence intensity was detected by dual-luciferase reporter system.

### 2.11. Rescue Assay

Cells were seeded in 24-well plate with group settings: pcDNA3 + pcDNA3 (0.6 *μ*g+0.4 *μ*g), pcDNA3 + pTGF*β*1 (0.6 *μ*g+0.4 *μ*g), and pTGF*β*1 + psh PTEN (0.6 *μ*g+0.4 *μ*g). Liquid A: 1 *μ*g of the plasmid was added and gently mixed into 50 *μ*L serum-free culture medium with opti-MEM. Liquid B: 1.5 *μ*L liposomal lipofectamine 2000 reagent was added and gently mixed into 50 *μ*L opti-MEM in room temperature for 5 min. Solution B was slowly added into liquid A and gently mixed and let at room temperature for 20 min.

### 2.12. iTRAQ Labelled Liquid Chromatography Tandem-Mass Spectrometry (LC-MS/MS) Analysis

An agilent multiple affinity removal lc column was operated in human 14/mouse3 affinity column. Following 12.5% SDS-PAGE electrophoresis (constant current 14 mA, 90 min), samples were stained with Coomassie blue. The iTRAQ labeling kit (AB SCIEX, USA) was applied for isotopically labeled samples. The chromatographic separated samples were analyzed by MS using a Q-Exactive mass spectrometer.

### 2.13. Methylation-Specific PCR (MSP) and Bisulfite Sequencing PCR (BSP) Analysis of TGF*β*1 Gene

A mix of 130 *μ*L CT conversion reagent was added for every 20 *μ*L DNA of samples. The mixture was placed on a PCR instrument for MSP reaction. The MSP nonmethylated primer (*U*) and the methylated primer (*M*) primers were designed online. The 1-3 mL sample with 250 *μ*L proteinase *k* was put into a 15 mL centrifuge tube for centrifugation at 3500 rpm for 3 min, and the collected DNA was treated with sodium bisulfite. The band size and specificity of the PCR products were determined by 1.0% agarose gel electrophoresis, and the remaining products were purified and sequenced.

### 2.14. Methylated DNA Immunoprecipitation Sequencing (MeDIP-seq)

Cells were treated with 1% formaldehyde so that the interbinding of DNA and proteins was fixed by crosslinking. Then, genomic DNA were interrupted by sonication to 100–500 dp fragments. The DNA fragment end repair was performed using paired-end DNA Sample Prep Kit. Precipitation enrichment of genomic DNA was carried out using a 5 mC antibody from magnetic methylated DNA immunoprecipitation kit. Qualified libraries were used for illumina-Hi Seq 2000 sequencing.

### 2.15. Cell Proliferation Assay

Cell proliferation was determined by CCK-8 and EdU assay. For CCK-8 assay, after relevant stimulation, cells were cultured in 96-well plate for 24 h, 36 h, 48 h, 60 h and 72 h. Then, 10 *μ*L CCK-8 kit solution was added into culture medium for 1 h. The absorbance of each well at 450 nm was detected. For EdU assay, cells were cultured in 6-well plate and subjected to relevant stimulation for 48 h. Then, culture medium was changed with fresh culture medium containing 3 *μ*M EdU for 2 h. Following washing with PBS to remove excess EdU, cell nucleus were stained using DAPI. Results were observed and photographed under fluorescence microscopy.

### 2.16. Cell Apoptosis Assay

Cell apoptosis was detected using Annexin V-FITC/PI staining. After relevant stimulation, cells in each group were collected, washed with PBS and stained with 10 *μ*L Annexin V-FITC fluorescent probe for 15 min. Then, cells were stained with 5 *μ*L propidium iodide (PI) for 15 min. Following rinsed with PBS to remove excess dye, results were measured using flow cytometry. The excitation wavelength was 360 nm and the emission wavelength was 460 nm.

### 2.17. Cell Invasion Assay

Two-chamber transwell assay was performed to assess cell invasion. Transwell membranes were precoated with Matrigel overnight. After relevant stimulation, 1 × 10^5^ cells in 200 *μ*L FBS-free culture medium were seeded into upper chamber. DMEM-F12 medium containing 15% FBS was added into the lower chamber. Following incubation at 37°C for 48 h, cells in transwell membranes were rinsed with PBS and stained using 0.1% crystal violet solution. Results were photographed by an inverted microscope. Cells in each group were counted.

### 2.18. Wound Healing Assay

Cell migration was detected using wound healing assay. After relevant stimulation, 200 *μ*L pipette gun head was drawn perpendicular to the marker stroke on the cell culture side. Then, the scraped-removed cells were washed using PBS. Following incubation in DMEM-F12 medium supplemented with 2% FBS at 37°C for 48 h, results were photographed under inverted microscope at 0 h and 48 h. Cell-cell distances were measured using Image J software.

### 2.19. Statistical Analysis

All experiments were repeated three times. Data were analyzed by GraphPad Prism 9.0 software (GraphPad Software Inc., San Diego, CA, USA) and presented as mean ± standard deviation (SD). Difference between two groups was calculated by *t*-test and between more than two groups was calculated by one-way ANOVA. *P* < 0.05 indicated that the data had significant differences.

## 3. Results

### 3.1. 5-AZA-DC Intervention Influenced the Regulatory Effects of TGF*β*1 on DNMT1 and Target Genes in Neuroglial Cells Under Oxidative Stress

Firstly, TGF*β*1^OE^ or shTGF*β*1 was transfected into neuroglial HEB, HM, HM06, and SVGP12 cells. Results of western blot showed that TGF*β*1^OE^ transfection notably raised the protein level of TGF*β*1 in neuroglial cells (*P* < 0.05, Figure 1(a)), while shTGF*β*1 transfection reduced the protein level of TGF*β*1 in neuroglial cells (*P* < 0.05, Figure 1(b)). HEB cells were subjected to Ang-1 and APOE4 genes knockout, as well as oxyglucose deprivation/reoxygenic stimulation, the mRNA expressions of DNMT1, TGF*β*1, PTEN, and TSC2 in HEB cells after TGF*β*1^OE^ (or shTGF*β*1) transfection and 5-AZA-DC treatment were measured. Results in Figure 1(c) displayed that both TGF*β*1^OE^ and shTGF*β*1 transfection raised the DNMT1 mRNA expression in HEB cells (*P* < 0.05), while 5-AZA-DC treatment reversed the effect of TGF*β*1^OE^ or shTGF*β*1 transfection on DNMT1 mRNA expression. 5-AZA-DC treatment notably enhanced the TGF*β*1 mRNA expression in TGF*β*1^OE^-transfected HEB cells (*P* <0.05). Both TGF*β*1^OE^ and sh TGF*β*1 transfection reduced the PTEN and TSC2 mRNA expressions in HEB cells (*P* <0.05), 5-AZA-DC treatment raised the PTEN and TSC2 mRNA expressions in HEB cells (*P* < 0.05). Results of western blot showed similar results in protein levels of DNMT1, TGF*β*1, PTEN, and TSC2 in HEB cells (*P* < 0.05, Figure 1(d)). These results suggested that 5-AZA-DC intervention influenced the regulatory effects of TGF*β*1 on DNMT1 and target genes in neuroglial cells under oxidative stress.

### 3.2. 5-AZA-DC Intervention Affected the Binding Between TGF*β*1 and PTEN Gene

The interactions between TGF*β*1 and PTEN (or TSC2) in HEB cells were determined by GST-pull down. Results in Figure 2(a) illustrated that TGF*β*1 interacted with PTEN and TSC2 in HEB cells. CHIP assay was applied for verifying the direct binding effect between transcription factor TGF*β*1 and target gene PTEN. Total chromatin input was used as a positive control and chromatin precipitated with IgG was used as a negative control. As shown in Figure 2(b), TGF*β*1 significantly enriched the target gene PTEN compared with normal rabbit IgG in HEB, HM, HM06, and SVGP12 cells, which indicated that TGF*β*1 can bind directly to the target gene PTEN. The influence of TGF*β*1^OE^ (or shTGF*β*1) transfection and 5-AZA-DC intervention on binding relationship between TGF*β*1 and target gene PTEN was detected. Results displayed that 5-AZA-DC intervention notably promoted the combination between TGF*β*1 and target gene PTEN in both TGF*β*1^OE^ (or shTGF*β*1) transfected neuroglial cells (P < 0.05, Figure 2(c)). Dual-luciferase reporter assay was utilized for confirming the transcription factor TGF*β*1 regulates PTEN promoter activity. pGL3-PTEN-luc, pGL3-Control-luc, and positive control plasmid pGL3-Basic-luc, were transfected into HEB, HM06, HM, and SVGP12 cells. Proteins were lysed 24 h after transfection and the intensity of luciferase was detected. Results showed that the fluorescence intensity of the cells transfected pGL3-Basic-luc, was significantly lower than cells transfected pGL3-PTEN-luc (*P* < 0.05, Figure 2(d)), indicating that TGF*β*1 bound to the promoter of PTEN gene. These results suggested that 5-AZA-DC.

### 3.3. 5-AZA-DC Intervention the Modulation of TGF*β*1 on PTEN Promoter Activity and Quantitative Proteomic Analysis of LC-MS/MS

To verify whether TGF*β*1 can regulate PTEN promoter activity, HEB, HM06, HM, and SVGP12 cells were subjected to shTGF*β*1 (or TGF*β*1^OE^) transfection and 5-AZA-DC intervention. Results showed that the promoter activity of PTEN was higher in the TGF*β*1^OE^ group and lower in the shTGF*β*1 group, compared to control group (*P* < 0.05, Figure 3(a)). 5-AZA-DC intervention further accelerated the promoter activity of PTEN in both TGF*β*1^OE^ and shTGF*β*1 groups (*P* < 0.05). To demonstrate that PTEN is a functional target gene of TGF*β*1, rescue experiment was designed. HEB cells were grouped as follows: pcDNA3 + pcDNA3, pcDNA3 + pTGF*β*1, and pTGF*β*1 + psh PTEN. Whether the exogenous knockdown of PTEN could rescue the low endogenous PTEN expression induced by TGF*β*1 in HEB cells were detected. Results displayed that the mRNA and protein expression levels of PTEN in the above three groups using real-time PCR and western blot analysis. Overexpression of TGF*β*1 promoted the endogenous PTEN mRNA and protein expressions, while endogenous PTEN expression levels were rescued after exogenous PTEN knockdown, indicating that exogenous PTEN knockdown can rescue the promoting effect of TGF*β*1 on PTEN expression (*P* < 0.05, Figure 3(b)). Following shTGF*β*1 (or TGF*β*1^OE^) transfection and 5-AZA-DC intervention, HEB cell quantitative proteomic diagnostic ROC independent indicator was analyzed. Results displayed that 5-AZA-DC intervention altered the proteomic diagnostic ROC independent indicator of HEB cells (Figure 3(c)). Quantitative proteomic analysis of the LC-MS/MS combination of HEB cells using iTRAQ technology found that there were 175 proteins were quantitatively identified. Further in-depth analysis showed that 44 proteins were significantly differentially expressed, of which 19 proteins were upregulated and 25 proteins were downregulated (Figure 3(d)). These findings suggested that.

### 3.4. MSP, BSP Detection and Methylated DNA Immunoprecipitation Sequencing (MeDIP-seq)

HEB cell lines had a relatively low expression of PTEN. The methylation status of PTEN promoter in HEB cells before and after 5-AZA-DC intervention was examined using the MSP technology. Results display that TGF*β*1^OE^ caused a significant increase in the DNA demethylation level of PTEN promoter, this indicated that TGF*β*1 inhibited the DNA methylation level at the PTEN promoter (Figure 4(a)). After sequencing through the BSP amplification, results found that PTEN gene was hypermethylated in HEB cells. BSP sequencing verified the results of MSP methylation analysis. Methylation was significant in the shTGF*β*1 and TGF*β*1^OE^ groups before the 5-AZA-DC intervention, and it was non-methylated after the 5-AZA-DC intervention (Figure 4(a)). About half of the promoter region contains CpG, and DNA methylation of the promoter region of CpG is again frequently associated with the transcriptional activity of the genes. We found consistent heatmap results and whole gene level for clustering analysis of promoter regions and CGI regions of these genes. In addition, considering that the CpG islands of the TGF*β*1, PTEN, and TSC2 genes are located in the promoter region, the methylation of the CpG islands causes a significant downregulation of TGF*β*1, PTEN, and TSC2 genes. Heatmap of the clustering of the gene promoter regions and the CpG island regions with the most distinct differences between the different groups of the HEB cell lines before and after 5-AZA-DC intervention were shown in Figure 4(b). Number of genes changing expression levels in differentially significant genes before and after 5-AZA-DC intervention was illustrated in Figure 4(c).

### 3.5. TGF*β*1^OE^ (or shTGF*β*1) Transfection and 5-AZA-DC Intervention Modulated Neuroglial Cell Proliferation and Apoptosis Under Oxidative Stress

Following TGF*β*1^OE^ (or shTGF*β*1) transfection and/or 5-AZA-DC intervention, neuroglial HEB, HM06, HM, and SVPG12 cells proliferation and apoptosis were tested. Results in Figure 5(a) showed that in groups of cells without 5-AZA-DC intervention, TGF*β*1^OE^ and shTGF*β*1 transfection reduced neuroglial cell proliferation (*P* < 0.05, Figure 5(a)). 5-AZA-DC intervention treatment raised the proliferation of HEB, HM06, HM, and SVPG12 cells (*P* < 0.05). Similar results were found in EdU incorporation assay, which showed that compared to HEB cells subjected to TGF*β*1^OE^ (or shTGF*β*1) transfection without 5-AZA-DC intervention, cells with 5-AZA-DC intervention had higher proliferative activity (*P* < 0.01, Figure 5(b)). Annexin V-FITC/PI staining was used to assess cell apoptosis. Results illustrated that both TGF*β*1^OE^ and shTGF*β*1 transfection accelerated HEB, HM06, HM, and SVPG12 cell apoptosis (Figure 5(c)). 5-AZA-DC intervention reduced cell apoptosis caused by TGF*β*1^OE^ or shTGF*β*1 transfection (*P* < 0.05). The results of Tunel assay showed similar tendency, which also displayed that TGF*β*1^OE^ and shTGF*β*1 transfection promoted neuroglial HEB cell apoptosis (Figure 5(d)), while 5-AZA-DC intervention lowered HEB cell apoptosis (*P* < 0.05). These results suggested that TGF*β*1^OE^ (or shTGF*β*1) transfection and 5-AZA-DC intervention took part in the modulation of neuroglial cell proliferation and apoptosis under oxidative stress.

### 3.6. TGF*β*1^OE^ (or shTGF*β*1) Transfection and 5-AZA-DC Intervention Modulated Neuroglial Cell Migration and Invasion Under Oxidative Stress

After TGF*β*1^OE^ (or shTGF*β*1) transfection and/or 5-AZA-DC intervention, neuroglial HEB cells invasion and migration were also tested. Results in Figures 6(a) and 6(b) showed that in groups of HEB cells without 5-AZA-DC intervention, TGF*β*1^OE^ and shTGF*β*1 transfection inhibited HEB cell invasion and migration. 5-AZA-DC intervention promoted HBE cell invasion and migration (*P* < 0.05). These results suggested that TGF*β*1^OE^ (or shTGF*β*1) transfection and 5-AZA-DC intervention also took part in the modulation of neuroglial cell invasion and migration under oxidative stress.

## 4. Discussion

Oxidative stress refers to the imbalance of oxidation and antioxidant effects [1]. Clinical oxidative stress is common in neurological diseases such as craniocerebral injury, cerebrovascular diseases, intracranial infection, intracranial tumors, and systemic diseases such as severe pneumonia and toxic dysentery [14–16]. Earlier, literature displayed that oxidative stress could cause intracranial hypertension, affect the blood perfusion of the brain, and even form a brain hernia and pathogenic death [17]. The occurrence of oxidative stress is associated with abnormal blood supplement in the brain and can cause brain cell dysfunction [18]. Our results confirmed that DNMT1 expression was significantly higher in oxidative stress neuroglia cells than normal neuroglial cells. TGF*β*1 expression had contrary phenomenon, which was lowly expressed in neuroglial cells than normal neuroglial cells. DNMT1 and TGF*β*1 expressions were significantly downregulated by methylation inhibitor 5-AZA-DC treatment, indicating that the expression of DNMT1 and TGF*β*1 expression are regulated by DNA methylation. Moreover, we found that significant methylation of the promoter of the transcription factor TGF*β*1 occurred in neuroglial cells after oxidative stress, which significantly affected the methylation level of the target gene PTEN and TSC2 after 5-AZA-DC intervention. The proposed signaling pathway was displayed in Figure 7.

TGF*β*1 is a protein about 92 kDa with multiple regulatory function in cell proliferation, death, migration, and differentiation [19]. The absence of PTEN causes intracellular PIP3 accumulation, imbalance the PTEN-PI3K/AKT signaling transduction pathway, and sustained AKT activation, further activating the mammalian target of rapamycin (mTOR) [20, 21]. With a molecular weight of approximately 200 kDa, mTOR hyperactivation caused by inactivation of TSC2 gene mutation is believed to be one of the causes of brain edema [22]. In the TGF*β*1/PI3K/PTEN/AKT/TSC2/mTOR cell signaling pathway, PI3K can activate its downstream signaling molecules to produce procell proliferation and antiapoptotic effects [23]. Activated Akt will further phosphorylate a variety of transcription factors and regulates which regulates cell survival, cell proliferation, and apoptosis [24]. The experimental results of this study confirmed that TGF*β*1 is involved in the regulation of biological functions such as neuroglial cell proliferation and apoptosis, suggesting that TGF*β*1 may participate in the pathogenesis of oxidative stress, and that its abnormal expression may be correlated with the biological dysfunction of neuroglial cells. We demonstrated that downregulation of TSC2 expression causes mTOR activation and the activated TGF*β*1 binds to promoter of PTEN gene to regulate PTEN expression at the transcriptional level. However, the molecular mechanism by which mTOR activates TGF*β*1 is not clear. More investigations are still needed in the future. In addition, our results showed that in the PI3K/PTEN/AKT/mTOR signaling pathway, AKT activity is regulated by PTEN genes located upstream and TSC2 genes located downstream, respectively. Increased CpG island methylation level in the promoter region of a gene will affect the gene transcription, and then inhibit the gene expression level and function, while demethylation can induce the gene expression and reactivation [25].

Previous literature discovered that TGF*β*1 may act as an important negative regulator in early oxidative stress development in regulating neuroglial cell proliferation and apoptosis, and this regulatory effect may be achieved by directly or indirectly regulating the activity of PTEN and TSC2 [26]. The application of a negative control group as a reference in our study to clarify the significance of the upregulation and downregulation of TGF*β*1 gene expression. We found that the demethylated drugs could increase TGF*β*1 mRNA expression in neuroglial cells, improve cell proliferation ability, and significantly inhibit cell apoptosis by changing the methylation status of the promoter region of the TGF*β*1 gene. Besides, we confirmed that DNMT1 expression was significantly higher in *in vitro* edema neuroglial cells than normal counterparts, and TGF*β*1 expression was significantly lower than in normal neuroglial cells. DNMT1 expression was significantly downregulated by the methylation inhibitor 5-AZA-DC treatment, indicating that the expression of TGF*β*1 is regulated by DNA methylation.

Earlier research demonstrated that TGF*β*1 was involved in the regulation of biological functions such as neuroglial cell proliferation, apoptosis migration, and invasion [27]. Herein, the influences of TGF*β*1 overexpression (or silence) and/or 5-AZA-DC treatment on neuroglial cell proliferation, apoptosis migration, and invasion were explored. We revealed that under oxidative stress, both TGF*β*1 overexpression and silence inhibited neuroglial cell proliferation, migration, and invasion, as well as promoted cell apoptosis. 5-AZA-DC treatment alleviated neuroglial cell proliferation, migration, and invasion inhibition and apoptosis caused by TGF*β*1 overexpression or silence. These findings suggest that neuroglial cell DNA methylation can significantly inhibit cell proliferation, migration, and invasion, as well as promote cell apoptosis.

MSP and BSP assays were applied in this research to examine the DNA methylation levels of DNMT1, TGF*β*1, PTEN, and TSC2 genes in neuroglial cells after oxidative stress. Neuroglial cells from oxidative stress brain edema showed upregulated methylation levels, and DNMT1 genes showed hypermethylation, while TGF*β*1, PTEN, and TSC2 genes showed hypomethylation. Therefore, we concluded that the oxidative stress regulation may be one of the important factors aggravating the DNA methylation levels in neuroglial cells. In *in vitro* cytology studies, we applied the methyltransferase inhibitor 5-AZA-DC intervention to treat neuroglial cells. We found that 5-AZA-DC took part in the modulation of multiple neuroglial cell functions. We considered that 5-AZA-DC improved the biological function of neuroglial cells under oxidative stress.

## 5. Conclusion and Perspective

In conclusion, we demonstrated that methyltransferase inhibitor 5-AZA-DC intervention inhibited DNMT1 activity, demethylated the promoters of TGF*β*1, PTEN, and TSC2 genes, thereby upregulated the expression of TGF*β*1, PTEN, and TSC2 genes in neuroglial cells under oxidative stress. It also participated in the regulation of neuroglial cell proliferation, migration, invasion, and apoptosis under oxidative stress. The findings of this study clearly revealed the protective effect of 5-AZA-DC on neuroglial cell under oxidative stress, providing a new idea and target for the potential therapeutic intervention method. More *in vivo* and clinical research are still needed to further explore the validity of 5-AZA-DC intervention on neuroglial cell oxidative damage in the future. We speculate that 5-AZA-DC may have important effects on the functional regulation of oxidative stress in neuroglial cells, it also provides a new experimental basis and intervention target for using epigenetic methods to study the treatment mechanism of oxidative stress.

## Figures and Tables

**Figure 1:** 5-AZA-DC intervention influenced the regulatory effects of TGF*β*1 on DNMT1 and target genes in neuroglial cells under oxidative stress. (a, b) The protein expressions of TGF*β*1 in neuroglial HEB, HM, HM06, and SVGP12 cells after TGF*β*1^OE^ or shTGF*β*1 transfection were determined by western blot. (c, d) HEB cells were subjected to oxyglucose deprivation/reoxygenic stimulation. The mRNA and protein expressions of DNMT1, TGF*β*1, PTEN, and TSC2 in cells after TGF*β*1^OE^ (or shTGF*β*1) transfection and/or 5-AZA-DC treatment were determined by real-time PCR and western blot. Data are shown as mean ± SD. ns: nonsignificant, ^∗^*P* < 0.05.

**Figure 2:** 5-AZA-DC intervention affected the binding between TGF*β*1 and PTEN gene. (a) The interactions between TGF*β*1 and PTEN (or TSC2) proteins were determined by GST-pull down assay. (b) CHIP was utilized to further verify the direct binding effect between TGF*β*1 and PTEN gene. (c) Cells were subjected to oxyglucose deprivation/reoxygenic stimulation. The interaction between TGF*β*1 and PTEN gene was detected using CHIP assay after TGF*β*1^OE^ (or shTGF*β*1) transfection and/or 5-AZA-DC treatment. (d) Dual-luciferase reporter assay was used to verify the binding between transcription factor TGF 1 and PTEN promoter. Data are shown as mean ± SD. ns: nonsignificant, ^∗^*P* < 0.05, ^∗∗^*P* < 0.02, ^∗∗∗^*P* < 0.01.

**Figure 3:** 5-AZA-DC intervention the modulation of TGF*β*1 on PTEN promoter activity and quantitative proteomic analysis of LC-MS/MS. (a) Following shTGF*β*1 (or TGF*β*1^OE^) transfection and/or 5-AZA-DC intervention, the promoter activity of PTEN was measured. (b) HEB cells were subjected to pcDNA3 + pcDNA3, pcDNA3 + pTGF*β*1, or pTGF*β*1 + psh PTEN transfection. After 5-AZA-DC intervention, the mRNA expression of PTEN in cells were detected. (c) Following shTGF*β*1 (or TGF*β*1^OE^) transfection and/or 5-AZA-DC intervention, the quantitative proteomic diagnostic ROC independent indicator was analyzed. (d) Results of quantitative proteomics analysis of iTRAQ-labeled LC-MS/MS. Data are shown as mean ± SD. ns: nonsignificant, ^∗^*P* < 0.05.

**Figure 4:** MSP and BSP detection, and MeDIP-seq. (a) The CpG island DNA methylation in the promoter region of PTEN gene was determined by MSP and BSP (b) Methylated DNA immunoprecipitation sequencing (medip-seq). (c) Number of differentially significant genetic changes before and after the 5-AZA-DC intervention.

**Figure 5:** TGF*β*1^OE^ (or shTGF*β*1) transfection and 5-AZA-DC intervention modulated neuroglial cell proliferation and apoptosis under oxidative stress. Cells were subjected to TGF*β*1^OE^ (or shTGF*β*1) transfection and/or 5-AZA-DC intervention, (a, b) cell proliferation was assayed by CCK-8 and EdU incorporation assay. (c, d) cell apoptosis was determined by flow cytometry and Tunel staining. Data are shown as mean ± SD. ns: nonsignificant, ^∗^*P* < 0.05.

**Figure 6:** TGF*β*1^OE^ (or shTGF*β*1) transfection and 5-AZA-DC intervention modulated neuroglial cell migration and invasion under oxidative stress. HEB cells were subjected to TGF*β*1^OE^ (or shTGF*β*1) transfection and/or 5-AZA-DC intervention, (a) cell invasion was determined by two-chamber transwell assay (magnification, ×200; scale bar = 20 *μ*m). (b) cell scratch assay was applied for measuring cell migration (magnification, ×200; scale bar = 40 *μ*m). Data are shown as mean ± SD. ns: nonsignificant, ^∗^*P* < 0.05.

**Figure 7:** The graphic overview of this research. 5-AZA-DC took part in the regulation of the effects of TGF*β*1 on target genes in neuroglial cells; thereby influence cell proliferation, apoptosis, migration, and invasion under oxidative stress.

**Table 1:** List of interference sequences.

Gene	Location	Sequences
Sh-TGF*β*1	110-168	GCATCTTCTTCGTGTTCAA
Sh-control	102-155	GCATCTCCATCGAAGGCTT

**Table 2:** Primers used for real-time PCR.

Primer set	Sequence	PCR product (bp)
DNMT1		
Sense	5-AGATGTGGATCAGCAAGCA-3	119
Antisense	5-GCGCAAGTTAGGTTTTGTCA-3	
TGF*β*1		
Sense	5-ACCCAACAGCCGCCGTAG-3	143
Antisense	5-CAGACTGGTTGTTTCCATTCAGAT-3	
PTEN		
Sense	5-CGACGGGAAGACAAGTTCAT-3	125
Antisense	5-AGGTTTCCTCTGGTCCTGGT-3	
TSC2		
Sense	5-CACTGGTGAGGACGTCTG-3	131
Antisense	5-CCGCAGCATCAGTGTGTC-3	
*β*-Actin		
Sense	5-AGATGTGGATCAGCAAGCA-3	87
Antisense	5-GCGCAAGTTAGGTTTTGTCA-3	

## Data Availability

The datasets used and/or analyzed during the current study are available from the corresponding authors upon reasonable request.

## Abbreviations

TGF*β*1: Transforming growth factor-*β*1
PTEN: Phosphatase and tensin homolog deleted on chromosome ten
TSC2: Tuberoussclerosis2
5-AZA-DC: 5-aza-2'-deoxycytidine
Ang-1: Angiopoietin-1
ApoE4: Apolipoprotein E4
DNMT1: Recombinant DNA methyltransferase 1
PI3K: Phosphoinosiol-3-kinase
AKT: Threonine protein kinase
mTOR: Mammalian target of rapamycin
FBS: Fetal bovine serum:
MSP: Methylation-specific PCR
BSP: Bisulfate-sequencing PCR
CCK-8: Cell counting kit-8
EDU: 5-ethynyl-2' -deoxyuridine
CHIP: Chromatin immunoprecipitation
LC-MS/MS: Liquid chromatography–tandem mass spectrometry.
